The article "Water, land, and air: how do residents of Brazilian remote rural territories travel to access health services?" was published in 2022. Journal: Arch Public Health.

# Water, land, and air: how do residents of Brazilian remote rural territories travel to access health services?

**DOI:** 10.1186/s13690-022-00995-z

**Published:** 2022-11-22

**Authors:** Patty Fidelis de Almeida, Adriano Maia dos Santos, Lucas Manoel da Silva Cabral, Eduarda Ferreira dos Anjos, Márcia Cristina Rodrigues Fausto, Aylene Bousquat

**Affiliations:** 1 Collective Health Institute, Federal Fluminense University - Niterói, Rio de Janeiro, Brazil; 2 Multidisciplinary Health Institute, Federal University of Bahia - Vitória da Conquista, Bahia, Brazil; 3 Institute of Social Medicine, State University of Rio de Janeiro, Rio de Janeiro, Brazil; 4 National School of Public Health Sergio Arouca, Oswaldo Cruz Foundation, Rio de Janeiro, Brazil; 5 Public Health Faculty, University of São Paulo, São Paulo, Brazil

**Keywords:** Transport, Health services accessibility, Public Health, Health disparities, Rural population, Brazil

## Abstract

**Background:**

Ensuring adequate and safe means of travel is essential for maintaining and improving the health and well-being of residents of rural communities worldwide. This article maps costs, distances, travel times, and means of elective and urgent/emergency health transport in Brazilian remote rural municipalities.

**Methods:**

Multiple case studies were conducted in 27 remote rural municipalities using a qualitative method. A total of 178 key informants (managers, doctors, and nurses) were interviewed. Secondary data from national information systems were analyzed for the socioeconomic characterization, to identify the costs, distances, and travel times. Through the thematic content analysis of the interviews, the means of transport, and strategies developed by managers, professionals and users for their provision were identified.

**Results:**

The costs of traveling between remote rural municipalities and locations where most of specialized and hospital services are centered can compromise a significant part of the families’ income. The insufficiency, restriction of days, times, and routes of health transport affects the selection of beneficiaries based on socioeconomic criteria in places of high vulnerability and less investment in road infrastructure. In remote rural municipalities, travelling to seek health care involves inter-municipal and intra-municipal flows, as their territories have dispersed populations. Several means of transport were identified – air, river, and land – which are often used in a complementary way in the same route. Some patients travel for more than 1000 km, with travel times exceeding 20 h, especially in the Amazon region. While the demands for urgent and emergency transport are partially met by national public policy, the same is not true for the elective transport of patients. The impossibility of providing health transport under the exclusive responsibility of the municipalities is identified.

**Conclusions:**

For the remote rural municipalities populations, the absence of national public policies for sufficient, continuous, and timely provision of transport for health services worsens the cycle of inequities and compromises the assumption of the universal right to health care.

## Background

The difficulties in accessing health services are expressed in various ways and affect different populations unequally. In addition, to measures aimed at providing it, policies and actions that will improve the needs and demands of the users, including transport to health services, are necessary [1]. Ensuring adequate and safe means of transport is essential for the maintenance and improvement of the health and well-being of residents of rural communities worldwide. It can minimize the problems associated with long distances one of the major factors affecting access to health services [2]. The absence of or insufficient means of transport can delay continuous access to health services, medications, reassessment of therapeutic plans [3], and selection of the healthcare, with greater impacts on the monitoring of chronic conditions [4]. For diseases such as cancer, expenses associated directly and indirectly with treatment, such as transporting patients and caregivers not covered with health insurance to hospitals, comprise “financial toxicity” which has disastrous consequences for patients and their families [5].

The conditions, availability, and strategies for guaranteeing means of transport are different among countries, and the degree of implementation of public policies to mitigate barriers to accessing health services also differs. In the United States, an estimated 5.8 million people postponed their medical care in 2017 due to transport problems, with disproportionate impacts for the poorest individuals with chronic conditions, even after controlling for sociodemographic and health characteristics [4]. Previous studies reveal a strong association between inadequate transport in rural areas and unmet health needs among elderly patients [6]. In Peru, among people with disabilities, transport barriers were mentioned by 61% of the participants in a national survey, a percentage higher than the one found in relation to architectural barriers, and they are more significant in rural areas than in urban areas [7].

However, public policies, in general, seem to be guided by what Porter [8] called “tarmac bias,” despite the worse living conditions in rural, undeveloped, and impoverished areas. He argues that governments and civil society organizations could play an important role in the integration of off-road populations through the strengthening of local networks, with gains for local democracy, social equity, and improved livelihood conditions for rural populations [8]. In countries such as South Korea, demand-responsive transport and sharing transport models were recently introduced as part of broader policies to improve rural life [6]. In the United States, ride-sourcing services have been proposed as an alternative for the elective transport of patients with the potential to decrease insurance costs by reducing absenteeism, promoting greater adherence to treatments, higher bed turnover, and safer access, although the possibility of the provision in non-urban areas is not clear [4].

In Latin American countries, there are emerging studies on the relationship between transport, health care, and policies aimed at mobility, which, where they exist, are mainly aimed at urban environments [9]. Although inadequate public transport can amplify social segregation by restricting access to the labor market, education, health care, and culture in densely populated areas [9], its effect can be more severe for the rural populations.

In a study conducted in a state in the northeast region of Brazil, transport represented the highest indirect cost (not covered by the Unified Health System) involved in cancer treatment with 19.75% of the monthly minimum wage. This indicates a negative association when compared with users from the capital and rural areas [10]. A study that explored the geographic barriers of access to health services in rural areas of the semiarid region of the Northeast, based on the location of cisterns that cover low-income households, reveals that 53.5% of this population lives more than 5 km (Euclidean distance) from a Primary Care Unit (PCU), and over 60% lives at more than 10 km from hospital or emergency care services [11]. The availability of spatial data on families in extreme poverty is essential for developing intersectoral policies in the health and transport interface [11]. Consequently, policies and actions must be implemented to mitigate such barriers that sometimes prevent users from taking the most adequate health care, in a timely manner, conditioning worse clinical prognoses [5, 10].

The health transport subsystems are transversal to the Health Care Network and seek to facilitate flows and counterflows of people and products. Access to means of transport is strongly influenced by the availability of resources, especially in elective situations [12]. According to Mendes [12], this subsystem operates with primary actions in which the transport is from the residence or place of illness to a health service and secondary actions which involve transport between health services. The subsystem operates in two modules: a) elective transport related to known and scheduled events and b) urgent and emergency transport, concerned with unforeseen clinical situations.

This article focuses on the primary actions of the transport subsystem and the two modules. The objective is to map costs, distances, travel times, and means of elective and urgent/emergency health transport in Brazilian remote rural municipalities (RRM) [13]. We argued that the deleterious effects on the health of the most vulnerable populations, attributed to the barriers imposed by the insufficient and inadequate provision of health transport, have not been dealt with by national public health policies.

## Methods

### Study design and setting

The study of the multiple strategies to guarantee access of populations living in rural and remote areas in Brazil to health services is very timely and contributes to the dialogue with several other realities. After all, Brazil has the fifth largest territorial extension in the world, countless ecosystems, ranging from desert areas to the Amazon Forest; from conservation regions to areas heavily impacted by agribusiness and mining; in addition to having several traditional populations.

In Brazil, the definition of rural and urban municipalities gained a new typology in 2017 [13], in line with methodologies from the Organization for Economic Co-operation and Development and the European Union. For a broader study to analyze the organization of primary health care (PHC) in RRM in Brazil [14], of which this article is a part, the 323 municipalities classified as remote rural were grouped in six clusters.

These clusters were constructed based on the analysis of the use of the territory, identifying the different ways in which the Brazilian territory was socially and economically occupied. The study of Santos and Silveira [15], which proposed a Brazilian regional division in “4 Brazils”: the Concentrated Region (South and Southeast); the Region of Recent Peripheral Occupation; the Northeast; and the Amazon, served as a basis for this analysis. Initially, the RRM were plotted on the Brazilian map according to these “4 Brazils”, identifying the areas with the highest concentration of these municipalities. Afterwards, we analyzed their respective logics of inclusion in the economic arena and their main forms of interconnection with the others points of the territories (terrestrial or fluvial) based on data available on the IBGE (https://cidades.ibge.gov.br/brasil/) and the National Department of Infrastructure and Transport (http://www.dnit.gov.br/mapas-multimodais/mapasmultimodais) websites. The following were listed: the profile of economic activities; the composition of the Gross Domestic Product according to the different economic activities; dependence on government transfers; the Gross Domestic Product per capita; population density, and percentage of population participating in cash transfer programs. These variables were chosen for their importance in the analysis of rural and remote scenarios worldwide, expressing the reduction of population, the remoteness, and the economic capacity. The characterization of municipalities led to the design of 6 clusters named: *Matopiba; North Minas; Central-West; Semiarid; North Waters; and North Roads*. These six clusters show distinct spatial logics, agglutinating 97.2% (307) of the 323 RRM. In Fig. 1 it is possible to locate on the map the 6 clusters used in the study and their distribution across the 5 large regions of Brazil.

**Fig. 1:** Distribution and location of research clusters by large regions of Brazil, 2019

The sample of municipalities was selected intentionally from defined clusters. These clusters were composed of two or more municipalities corresponding to the "municipality type", that is, with socioeconomic, demographic, and health characteristics commonly found in the group of RRM of the respective cluster. One or more outlier municipalities were added to the municipality type, according to the same criteria, with more uncommon characteristics in the area. Thus, we sought to ensure the inclusion of different realities of the RRM, which allowed for an in-depth analysis of the constraints for the health system and the numerous strategies used by the population, professionals, and managers to guarantee access to health services. With this procedure, we obtained an intentional sample of 27 municipalities distributed in the six previously defined areas, in which multiple case studies were carried out, with a qualitative approach, based on interviews with key informants, complemented by secondary data from national information systems.

To understand the intramunicipal particularities, the territory was classified into two areas: the RRM headquarters, identified as the urban nucleus – where public facilities, commerce, and services, in general, are concentrated – and the rural area – a the “interior” area of the municipality that corresponds to small and dispersed population groups located in regions far from the headquarters.

### Participants and data collection

The study population comprised 178 respondents: municipal health managers – municipal health secretaries and PHC coordinators (53), regional managers (15) of each of the six health regions to which the 27 municipalities belonged, State PHC managers (12) in each of the states involved, and doctors and nurses from the PHC teams (98) of all municipalities (Table 1). The first group of key actors, composed of managers, are responsible for the management and organization of the Health Care Network in the Brazilian Unified Health System, which, according to the Brazilian federal system, establishes the public and universal provision of health services under the responsibility of the three spheres of government: federal, state, and municipal. The second group of informants comprised doctors and nurses who worked in a PCU at the headquarters and one in the rural area of ​​the selected 27 RRM, which are part of the teams of the Family Health Care Strategy. The Family Health Care Strategy is the main PHC model in the country and covers approximately 134 million inhabitants through 43,286 teams (Dec/2020) [16]. The teams are composed, necessarily, of doctors and nurses (in addition to community health workers and nursing technicians) who act as generalists gateway to other care services. In this sense, they are privileged informants in relation to the difficulty of access faced by users.

**Table 1:** Research participants by typology of territories and remote rural municipalities in Brazil, 2019

Participants	Central-West	Matopiba	North Waters	North Roads	North Minas	Semiarid
State Managers	1	3	4	1	1	2
Regional Managers	2	3	3	2	2	3
Municipal Health Managers / Primary Health Care Coordinators	5	14	15	5	6	8
Nurses	5	11	16	6	6	8
Doctors	5	9	14	4	6	8
**Total**	**18**	**40**	**52**	**18**	**21**	**29**

Source: Interview: “Primary Health Care in RRM in Brazil” (Fausto, 2020)

The interviews were based on multidimensional scripts to understand the organization and provision of PHC services and their relationship with other health services to ensure comprehensive and integrated care, in accordance with the objectives of the broader study [14]. The scripts were composed of general and specific dimensions, according to the type of person interviewed: characteristics of the territory and population served, PCU structure, access to PHC services, specialized and hospital care, health transport, work process, community participation, among others [4]. The analyses in this article focused on topics related to the means of elective and urgent/emergency health transport and actions developed in different scenarios of provision. The respondents were interviewed face-to-face at their respective workplaces by the project’s research team, from May to October 2019, with an average duration of 1:00 (doctors/nurses) to 2:30 h (managers), recorded in audio and transcribed in full.

Complementarily, data from national information systems were used to characterize the municipalities, costs, distances/times with displacement to seek health care.

### Data analysis

RRM context is an important component for understanding the magnitude of the access difficulties caused by the absence/insufficiency of policies for the provision of health transport. Key indicators were used for the often-unfavorable socioeconomic characterization of rural populations [8]. Secondary data were analyzed from three official national databases: Atlas of Human Development in Brazil, Brazilian Institute of Geography and Statistics (IBGE in Portuguese), and Ministry of Social Development referring the Panel of *Bolsa Família* Program and *Cadastro Único* of the beneficiary population of the *Bolsa Família* (Family Allowance Program—national income benefit program for people in extreme poverty), whose reference year is 2019.

The socioeconomic analysis is complemented by per capita income indicators and calculation of estimated costs and distances for travel: a) intra-municipal – from the rural area to the headquarters of the RRM; b) from the RRM to the headquarter municipality of the health region; c) from the RRM to the capital of the respective states. PHC services are often the only ones offered in the RRM, being responsible for referring patients to specialized and hospital services. Specialized and hospital services are usually offered in the municipalities that serve as headquarters of the health region or in the capitals of the respective states, through an agreement between managers of the Unified Health System. In all cases, health transport schemes are needed to enable access. We used information from the Strategic Maps for Citizenship Policies to identify the distance in kilometers for the routes a, b, and c. These maps allow the identification of the rural district with the greatest distance from the RRM headquarters (a) and provide access to information of the Highways Department of the States to define the distances between the 27 RRM and the respective headquarter municipalities of the health regions and capital (b, c). The ESRI ArcGIS PRO Georeferencing tool was used to measure the distances (kilometers) in straight lines between the municipalities/health regions/capital that have river roads, like those in the Amazon region.

After calculating the distances, the costs for traveling between routes a, b, and c were estimated based on the average annual gas price in Brazil (2019)—National Agency for Petroleum, Natural Gas, and Biofuel—and on the average consumption for land and river transport (National Institute of Metrology, Quality, and Technology), depending on the type of territory.

A thematic content analysis of the interviews was conducted. The means of health transport were classified into two modules for categorization purposes: a) elective transport – directed to known and schedulable events, whose key variable is timely, safe, and comfortable access to previously scheduled health services; b) urgency/emergency – clinical events not previously known, not scheduled, and that pose immediate risks [12]. The stages of thematic content analysis were: a) in-depth reading of the 178 interviews by pairs of researchers; b) selection, grouping and classification of excerpts with relevant structures and central ideas (thematic cores) in an analytical framework, based on previous categories; c) production of the various communication corpus, since the set of information was not homogeneous and emerged from different groups of subject representation (managers and PHC professionals) and clusters; d) subsequently, a comparison was made between the different participants of the research, in the confrontation of ideas and positions, having as reference the central objective of the study; e) to ensure the quality and validity of the findings, the information produced in the interviews and secondary data was crossed.

The analysis of interviews and secondary data complement each other by giving an idea of the dimension of geographic barriers to accessing health services and allowing the estimation of the travel distance/time. Information on the average travel time for some routes (not available from secondary sources), for example, was also obtained by the thematic analysis of the interviews. The intention was not the judgment of each municipality but the understanding of processes in the six territories.

Along with the mapping of means of transport, we identified strategies and actions taken by managers, users, and professionals to reduce the barriers arising from the absence or insufficient guarantee of health transport, which are greater in rural territories, as identified in other studies [2, 4, 5].

### Ethics approval

The study followed the ethical procedures approved by the Ethics Committee for Research in Human Beings of the Sérgio Arouca National School of Public Health of the Oswaldo Cruz Foundation (Nº 2.832.559). All participants signed the Informed Consent Form prior to participation.

## Results

### Context of RRM: socioeconomic characteristics and costs of transports

Table 2 presents socioeconomic indicators that are necessary to understand the living conditions in RRM. The national standard and the percentage of the population in extreme poverty and those who are beneficiaries of the federal program that we used as reference show the extreme vulnerability of the cases. The national Gini Index shows the great inequality of income in Brazil. The smaller Gini Index in 18 of the 27 RRM does not indicate greater equality, but only a generalized distribution of poverty. Likewise, the low Municipal Human Development Index of most cases confirms the set of vulnerabilities to which populations in remote rural territories are exposed. Some municipalities have higher values of Gross Domestic Product per capita due to agribusiness and mining activities. Low demographic density, with small and dispersed populations (only in 6 cases with a population above 20 thousand inhabitants), is also a characteristic of the RRM, with important implications for intra and intermunicipal transport.

**Table 2:** Socioeconomic indicators in Remote Rural Municipalities, Brazil, 2019

Territories	Country/ Municipality		State	Population ^a^	Per capita GDP ^b^ *(US$*^*c*^*)*	Demographic density^d^. (pop./km^2^)	Gini Index ^d^	MHDI^d^	% pop. extreme poverty ^d^	% beneficiary population PBF^e^
Central-West	**Brazil**			**210,147,125**	**8,110.70**	**23.8**	**0.60**	High	**6.62**	**21**
	Nova Lacerda		MT	6,640	6,699.08	1.32	0.51	Medium	12.90	31.15
	Tabaporã		MT	9,489	10,544.18	1.10	0.44	Medium	5.54	12.82
	Vila Bela da Santíssima Trindade		MT	16,128	4,792.22	1.16	0.59	Medium	15.10	25.37
Matopiba	Avelino Lopes		PI	11,289	1,696.78	8.81	0.56	Low	32.35	89.04
	Campos Lindos		TO	10,116	7,462.56	3.02	0.67	Low	31.11	34.28
	Formosa da Serra Negra		MA	19,089	1,787.62	5.15	0.63	Low	57.83	58.32
	Júlio Borges		PI	5,627	1,857.29	4.27	0.53	Low	36.78	71.37
	Monte Alegre do Piauí		PI	10,613	4,463.45	4.32	0.57	Low	30.39	59.70
	Redenção do Gurguéia		PI	8,778	2,033.69	3.50	0.57	Low	28.59	90.49
	Tasso Fragoso		MA	8,521	33,246.50	1.93	0.58	Low	27.43	56.04
North Waters	Aveiro		PA	16,388	1,741.61	0.93	0.60	Low	41.63	48.80
	Boa Vista do Ramos		AM	19,207	1,796.14	7.14	0.59	Low	40.05	52.16
	Curuá		PA	14,393	2,117.85	9.78	0.60	Low	38.99	62.18
	Maués		AM	63,905	1,928.86	1.56	0.64	Low	34.31	71.10
	Melgaço		PA	27,654	1,569.18	3.97	0.55	Low	43.92	81.12
	Prainha		PA	29,866	2,332.63	1.97	0.68	Low	42.48	75.23
	Vitória do Jari		AP	15,931	2,930.69	5.97	0.58	Medium	22.33	56.00
North Roads	Assis Brasil		AC	7,417	3,026.10	1.40	0.61	Low	30.66	75.98
	Jacareacanga		PA	41,487	12,523.54	0.15	0.69	Low	42.41	28.88
	Rurópolis		PA	50,510	1,708.94	6.99	0.57	Low	24.43	27.82
North Minas	Bonito de Minas		MG	11,230	1,498.67	2.78	0.57	Low	35.66	54.57
	Indaiabira		MG	7,351	1,907.11	7.49	0.48	Medium	13.97	56.98
	Rubelita		MG	5,995	2,179.29	6.11	0.50	Low	23.36	73.26
Semiarid	Ipupiara		BA	9,865	1,965.21	9.62	0.50	Low	23.79	62.93
	Morpará		BA	8,519	1,798.36	4.27	0.55	Low	29.89	80.52
	Pilão Arcado		BA	35,048	1,640.85	3.07	0.60	Low	40.90	65.46
	Rio Grande do Piauí		PI	6,432	1,893.06	9.95	0.54	Low	31.13	80.16

Source: ^a^ Population estimate, Brazilian Institute of Geography and Statistics (IBGE), reference 2019

^b^ Brazilian Institute of Geography and Statistics (IBGE), Gross Domestic Product—GDP, reference 2019

^c^ Dollar Exchange Rate in 2019: US$1.00 = R$4,1414, according to the Central Bank of Brazil

^d^ Municipal Human Development Index, Brazilian Institute of Geography and Statistics (IBGE), Demographic Census – (reference/2010). Note: Populations in extreme poverty are those with per capita income below US$ 13.21

^e^ MDS – Ministry of Social Development, *Bolsa Família* panel and *Cadastro Único*. Beneficiary population of the *Bolsa Família* Program (PBF—national income benefit program for people in extreme poverty), reference 2019

Table 3 shows that the monthly per capita income of families was less than US$100 (except in the Central-West). The table, based on the estimated expenditure on fuel by type of transport used (according to climate, geography, and condition of the roads), allows us to infer the magnitude of the impact on the income of families and individuals in the case of trips financed with their own resources, whether internal to the municipality itself (rural area-headquarters RRM) or the headquarter municipality of the health region or capital.

**Table 3:** Per capita income and estimated travel expenses, rural area—headquarters of the RRM – municipality headquarters of the health region—capital of the state, Remote Rural Municipalities, Brazil, 2019

**Territories**	**States**	**Gasoline/liter **^**a**^ (US$**)	**Municipality**^**b**^	**Per capita income **^**c**^ (US$**)	**Estimated expenses with travel:**		
					**RA- RRM**^**d,e**^** headquarters** (US$**)	**RRM- HR**^**d,e**^** headquarters** (US$**)	**RRM-Capital**^**d,e**^ (US$**)
Central-West	MT	1.14	Nova Lacerda	105.60	16.06	25.66	111.79
			Tabaporã	131.96	21.71	22.16	155.33
			Vila Bela da Sant. Trindade	106.04	28.77	15.11	101.29
Matopiba	TO	1.15	Campos Lindos	70.66	11.79	43.40	122.99
	MA	1.12	Formosa da Serra Negra	39.39	9.85	30.77	185.04
			Tasso Fragoso	63.93	14.66	27.51	181.77
	PI	1.13	Avelino Lopes	52.87	6.37	36.12	154.15
			Júlio Borges	43.37	11.01	39.21	157.43
			Monte Alegre do Piauí	65.49	13.52	29.56	147.78
			Redenção do Gurguéia	61.80	11.11	10.24	129.62
North Waters	AM	1.12	Boa Vista do Ramos^4^	42.39	268.32 *	67.08 *	402.47 *
			Maués	58.99	536.63 *	89.44 *	402.47 *
	AP	1.11	Vitória do Jari	74.71	132.71 *	11.46	64.89
	PA	1.18	Curuá	43.69	282.22 *	47.04 *	337.02
			Melgaço	32.65	353.89 *	24.33 *	398.13 *
			Aveiro	35.91	94.07 *	141.11 *	386.59
			Prainha	46.68	94.07 *	94.07 *	341.50
North Roads	PA	1.18	Rurópolis	58.55	36.78	44.22	323.03
			Jacareacanga	69.82	78.76	152.37	431.18
	AC	1.24	Assis Brasil	70.35	25.11	23.46	72.49
North Minas	MG	1.18	Bonito de Minas	47.24	30.15	9.63	129.25
			Indaiabira	68.28	6.35	18.09	146.14
			Rubelita	60.12	7.64	6.03	125.83
Semiarid	BA	1.13	Ipupiara	62.37	23.13	31.03	119.32
			Morpará	54.22	10.99	16.58	139.36
			Pilão Arcado	47.32	30.65	54.17	151.89
	PI	1.13	Rio Grande do Piauí	60.09	5.41	26.08	73.41

Caption: ^*^ Routes that are conducted by waterways

^**^ Dollar exchange rate in 2019: US$1.00 = R$4.1414. Source: Central Bank of Brazil

^a^ The average annual price of gasoline, per liter, in 2019 by Brazilian states. Source: National Agency of Petroleum, Natural Gas and Biofuels (ANP in Portuguese)

^b^ To measure fuel consumption on land routes, the average consumption of a car (pickup truck) with 4 × 4 traction was considered, which is a vehicle that is used in the six territories of the research. The average consumption, according to the National Institute of Metrology Standardization and Industrial Quality, is 5.85 km/liter. To measure fuel consumption on river routes, the average consumption was taken from the propulsion engine for motorboats, which include “*voadeiras*” and “*rabetas*” (outboard boats). The average consumption of this type of engine, according to the National Institute of Metrology Standardization and Industrial Quality, is 20 L of gasoline/hour

^c^ Brazilian Institute of Geography and Statistics (IBGE), Demographic Census – (reference/2010)

^d^ Strategic Maps for Citizenship Policies (MOPS) of the Ministry of Citizenship and Ministry of Women, Family and Human Rights—(Reference/2019)

^e^ Department of Roads and Highways (DER) of the states of Tocantins (TO), Maranhão (MA), Piauí (PI), Mato Grosso (MT), Minas Gerais (MG), Amazonas (AM), Amapá (AP), Pará (PA), Acre (AC), and Bahia (BA) – (Reference/2019)

### By water, land, and air: means of health transport in RRM

#### Elective health transport

The means of transport to access elective health services varied across municipalities and within them. The means used were identified for the following: a) transport to the PCU, specifically, by the populations of the rural area of the RRM and; b) specialized and hospital services provided in other municipalities and used by users in the RRM headquarters and rural areas. In both situations, the means of transport were provided by either the municipal administration or direct expense of users or their families.

As a common characteristic, none of the RRM studied have a structured logistic system for continuous and satisfactory provision of health transport. The transport routes, primarily by land, were often unpaved, especially in rural areas, and vehicles were insufficient, intermittent, and inadequate for the diversity of the population’s needs. Furthermore, the conditions of the roads and the distances to be covered increased the danger of some routes. With the use of motorcycles, the risk of accidents increased. In territories with populations mostly in conditions of a financial shortfall, the elective health transport system was required with considerable frequency and on a large scale due to characteristics intrinsic to the RRM and the location of specialized and hospital services, which were outside of the municipality of residence of the users.

All municipalities had some type of vehicle (minibuses, cars, vans, pickup trucks, boats, among others) funded with their own resources and, therefore, subject to discontinuities arising from budgetary limits and/or management capacity. The less complex municipal ambulances, although considered a modality of urgent and emergency transport, also attended to elective transport in some situation.

In any case, commonly, the provision of transport through municipal resources was primarily intended for users whose socioeconomic vulnerability prevented them from bearing the costs of traveling to health facilities, substantial portion of the population. In one of the cases, it was estimated that, due to the socio-economic conditions of the population, only one in ten residents would be able to pay for transport. In this sense, the funding and determination of priority for the selection of users, generally under the responsibility of the municipal administration, made this resource strongly crossed by clientelist interests.

Specifically, for users traveling to PCU, with rare exceptions, there was no provision of health transport, even to the most remote locations in the rural area of the RRM. Thus, the use of rides on school buses was a recurrent alternative in the territories. As such vehicles did not circulate during school holidays, the flow of users from the rural area to the PHC services located at the headquarters decreased. Another alternative for the residents in rural areas was to travel by foot or drive with their own resources – vehicle, river, animal – ride with neighbors and family members, or be even carried in hammocks with travel that could take up to two days. Aiming at a single cost of transport (outshopping), it was common for users in rural areas to seek health services when they went to the headquarters for other activities (to the bank, lottery stores, market). Thus, they optimize time and resources.

As there is no public transport in the rural area, there was a network of alternative transport for residents of the region, with increased values that compromised the families’ budget. In part of the municipalities where specialized consultations were in the state capital, users were instructed to go to the headquarters the day before on their own, from where the health transport departed. In this situation, it was common for users in rural areas to delay the search for care and seek assistance when affected by acute illnesses or worsening of chronic processes. Sometimes, they used alternatives present in informal subsystems, such as self-medication, teas, and medicinal plants, among others. However, in exceptional cases – bedridden people or people with specific health condition – it was possible to make a vehicle available by the municipal administration to travel from their residence to the health services. In addition, in rural areas, even the contact to request transport was difficult because of the lack of a telephone signal in some areas.

For specialized and hospital services located in other municipalities, the larger the territorial extension, the more was the difficulty in getting around, especially for residents of rural areas. To conduct consultations or specialized examinations, they made two trips to reach there (from the countryside to the RRM headquarters and then to the specialized/hospital services) and two trips to come back, which were sometimes considerably difficult. In some indigenous villages in North Roads, it took up to four days to reach the headquarters of the municipality (about 2000 km away).

In all studied RRM, for long-term treatments (hemodialysis, cancer), some means of transport was guaranteed for the user and a companion, regardless of the financial condition. In these cases, there were vehicles and/or commercial bus tickets paid for by a federal program called Treatment Outside the Home. Even then, the funding of this Program was still insufficient and was often supplemented by municipal resources. Larger vehicles such as vans, available in some wealthier municipalities, served to transport a greater number of users to the locations where continued care was provided.

In addition to the commonly used means, geographic, climatic, socioeconomic, and management specificities present in the RRM, and its territories conditioned various responses and strategies for the provision of means and modes of transport to access elective health services.

For travel to specialized care, in one of the RRM in the North Minas territory, there was a minibus managed by the Intermunicipal Health Consortium. This service, although more costly, was considered safer, as the Consortium was responsible for managing passengers and paying insurance in the event of an accident, which represented a certain amount of legal certainty for the administration. Cars offered by local merchants to the rural population for shopping at the municipality’s headquarters were also used to assist the PHC services.

In a municipality in the Semiarid region, the most viable option was to pay for tickets on intermunicipal buses, whose schedules did not always meet those made in other municipalities. Occasionally, it was “easier” to ensure transport to Salvador (state capital), where commercial buses left at night and arrived in the morning, merely in time for the consultation or examination. In these cases, it was necessary to ensure some type of support in the capital to assist in the mobility of users, especially those from rural areas.

In the Central-West area, the only territory in which all researched municipalities had an average Municipal Human Development Index, with lower percentages of *Bolsa Família* beneficiaries (Table 2). In this municipalities there seemed to be greater availability of cars, vans, and pickup trucks. Some of these were purchased through parliamentary amendments (federal and state public budget resources legally awarded to parliamentarians for public purposes) mainly to meet the demands of users in the rural area. These resources were used to return to the residence after traveling to the headquarters, travel to specialized services in other municipalities, and transport bedridden people. Such vehicles also served to support the activities of PHC teams, home visits, and sanitary and epidemiological surveillance actions. Therefore, they were not always available to transport users.

In the territory of Matopiba, no specifics were identified in relation to health transport (apart from municipal cars and some vans). It highlighted frequent reports of the administrations and professionals regarding their dependence on their own ambulances, especially on the SAMU (stands for “Mobile Emergency Care Service” in Portuguese) for the transport of users. There were reports of payment for intermunicipal buses for the most vulnerable users (the vast majority), especially in the municipalities belonging to the state of Piauí, which has its specialized health care units located mainly in the state capital.

In the North Waters territory, boats such as “*voadeiras*” and “*rabetas*” (small boats with outboard motors), regular boats and water ambulances were used due to geographic and climatic characteristics. In the isolated municipalities (Melgaço, Maués, and Aveiro), there were only cars and other means of land transport at the municipal headquarters. For other areas, only water transport was available. The use of both suffered variations due to extreme climatic conditions in the Amazon. Even municipalities that had public transport (circular buses) or ambulances (extremely frequent) experienced an interruption in circulation due to the need for repairs caused by the precariousness of the roads damaged by the rain. Transport was considered by respondents as the most critical resource for the provision of health services, with the high cost of fuel for river transport being highlighted (Table 3). Both ambulances (more complex structures for emergencies) and common river vehicles were used for elective transport of users; often, part of the route was completed by one or more means of land transport.

In the North Roads, which does not have a water ambulance, in case of trauma, the users themselves sought the service using “*voadeiras*.” In addition, many journeys by land were interrupted by precarious roads that became impassable (muddy roads) in the rainy season, increasing travel times, costs, and preventing the use of larger-scale transport such as buses. In RRM of North Waters and North Roads, the need for 4 × 4 traction cars and pickup trucks was reported due to road conditions, more frequently when compared to the other territories in the study.

Users of riverside communities in North Waters and North Roads, whose transport was by the river and who did not have boats or “*rabetas*,” depended exclusively on transport provided by the municipality or community support (relatives and neighbors). Another aspect was the lack of security, as there have been reports of accidents with women in small boats where several other users were traveling, in which women’s hair got stuck in the engine, and they ended up being scalped. For these populations, the Fluvial PCU was one of the ways to take assistance to places of difficult access, minimizing the problem of long distances. The Fluvial PCU was usually moored in central communities with a larger number of families and residents of adjacent communities coming to the vessel for service.

The acquisition of vehicles through resources of federal and state parliamentary amendments was a common procedure. Nevertheless, the cost of drivers, repairs for poor road conditions, and fuel was municipal. Such critical resources collaborated to the discontinuity of the provision of elective transport to the population.

In these cases, the use of vehicles from other sectors such as education, social assistance, and agriculture or requests from social assistance resources to pay for tickets for users and their companions were common.

The assessments of the difficulty in providing elective transport, either health transport or common transport, were unanimous. Occasionally, transport represented a greater challenge than the provision of the health service itself, with even more unfavorable differences for the dispersed population in the interior/rural areas of the RRM. Table 4 presents expressive statements by key respondents that show the challenges and arrangements for the provision of some means of health transport in the RRM. To maintain anonymity, respondents were identified by acronyms that correspond to their category and the state to which they belong, both related to the respective research territory.

**Table 4:** Summary of “expressive statements” about the challenges for access to health transport, Remote Rural Municipalities, Brazil, 2019

Territories	Elective and emergency transport	Expressive statements
Central-West	Ambulance purchased with parliamentary amendment resources	People, there is no such thing as refusing resources from the parliamentary amendment! Who wouldn't want the resources? We bought two ambulances with parliamentary amendment resources; therefore, the difference is to seek resources somehow. (1/RM/MT)
Matopiba	Intermunicipal bus	Users go on their own to Teresina (capital). Sometimes, we give them tickets. I spend ten thousand reais per month on transport. Many come to ask me because the price of the ticket is high, and they cannot afford it. We help many of them, more serious cases; for example, we have many cases of cancer. (1/MM1/PI)
	Municipal ambulances	We also have an ambulance that is here in the village, depending on the case of people who cannot move; in these specific cases, we will pick them up. (1/NUR/RA/MA)
North Waters	*Voadeiras* (small boats)	For Boa Vista do Cuçari, we have a *voadeira* that does not belong to the health services but is rented and contracted by the health services to transport patients to Monte Alegre. Santa Maria also has the *voadeira* that sends patients here, all offered for health services. (1/MM2/PA)
	Water ambulances	The riverside communities have difficulties of access because access is only by river, and not everyone has a canoe or boat available to get around… (…) So, sometimes, when the place has a telephone signal, they call, and we’ll go and pick them up. We have nine water ambulances in the rural area of the municipality and one water ambulance, equipped as if it were a bed, in the urban area; then there is the equipment that we take, a medicine box, and an oxygen box. (1/MM2/PA)
	Municipal and state ambulances	I do not know if there is a way to criticize that the ambulance here should be 4 × 4 traction. Most times, we send patients there, but the ambulance does not go because it does not move through the mud. Sometimes they come, but there are no conditions; they get halfway there, but they do not go beyond there if it is an urgent case. There are no conditions. (1/DOC/RA/PA)
North Roads	4 × 4 traction car	They called: “there’s a patient in a local area to go for an appointment or an emergency”. I asked, “does the ambulance get there?” “It does,” and off goes the ambulance. “No, the ambulance doesn’t get here,” off goes the pickup truck because there are places that even the pickup truck can’t reach; so, imagine a little ambulance… (2/MM2/PA)
	Car	The driver arrives earlier, he is experienced, but it usually takes four hours. Now imagine a patient with only an hour to live… there are some villages that are three days from here, and communities that take four to five hours by car; it can be some 200 km because the roads are bad. (3/MM2/PA)
	Airplane	Our biggest problem is the people involved in accidents, motorcycle, and car accidents. And each patient costs the municipality a range of R$15.000 to travel to Santarém, as it is by airplane. (1/MM1/PA) The airplane is private, and the city hall pays; they are small planes that are called “*teco-teco*”; when it is necessary and the patient is in serious condition, for example, we already had two mobile ICU transfers in this period now, the plane came fully equipped and with an intensivist, who performed the intubation and took the patient. (3/MM2/PA)
	Users carried in hammocks	When it rains, there are no conditions to reach the branches due to the amount of mud. Patients sometimes arrive carried in hammocks, as we have to have traction pickup trucks to be able to arrive and, many times, we cannot. The situation is very bad. (1/MM1/AC)
North Minas	Municipal ambulances	There are a lot of homes far away. I even suggested to a son, with a 90-year-old elderly woman, living in a place so far away; what if she gets sick? Don’t use the phone until he gets in touch with someone to arrange an ambulance… And the ambulance can’t get there, it’s a downhill, you go down and there’s only rock. No car can pass. (1/NUR/RA/MG)
	School bus	But most of the population uses transport linked to the city hall, like the school bus. They take the school bus that brings their daughters and goes to the primary care unit (located in the RRM headquarters). (1/MM2/MG) No [there is no public transport in this area]; there is only school transport that ends up giving people a ride. (2/NUR/RA/MG)
Semiarid	Cars from other areas—education and social assistance	And today, we don’t have money for transport; the transport that we have in health services can be counted on our fingers. We have a car that takes the doctor every day and another car that travels (for patients). And we end up using the education and social assistance car for health services. There are days when the three cars are on the road to take patients, go to appointments with specialists, or have an exam… (1/MM2/BA)
	Private cars paid by users	On average, the dentist sees from 5 to 7 people, but because of the rural area, we schedule to see at least 10 in the morning. And those 10 people come because if I schedule 5, they can’t come because of transport. There is a location here where the private car charges R$ 40,00 per person. So, if he manages to put 10 people in the service schedule, this price decreases. (2/MM2/BA)

Source: Interview: “Primary Health Care in RRH in Brazil” (Fausto, 2020)

Identification of respondents: municipality number/type of informant/state

*RM* Regional Manager, M*M1* Municipal Health Secretary, *MM2* PHC municipal coordinator, *NUR* Nurse of the PHC team, *DOC* PHC team doctor, *RA* Rural area

#### Urgent/emergency transport

The municipalities, roughly speaking, had logistics solutions through adequate vehicles to stabilize and/or reverse the troubling situation intended for the transport of people in urgent and emergency cases.

The major means of transport for emergencies is the SAMU of a regional nature. The SAMU, financed through federal and state resources, has mobile prehospital care, with services authorized by doctors in regional regulatory centers located in some municipalities, comprising the State Urgent and Emergency Networks.

For political reasons, not necessarily health ones, some managers wanted to have the SAMU headquarters in the municipality itself, as they considered that they would have easier access to ambulances, although some acknowledged that there was no necessary structure for that. In general, the SAMU ambulances met the needs of the headquarters, with greater difficulties in serving rural areas. For areas with restricted access, the combination between common and adapted transport that move patients to a SAMU ambulance was prevalent, reducing travel time. In some territories, during rainy seasons, residents often do not have access to the SAMU, which, together with PHC professionals, improvised transport in more serious cases.

The municipalities also had their own ambulances, which were less complex but often could not travel along the local roads, roads without pavement, and muddy or drought (sand) roads. It was suggested that ambulances should also have four-wheel drive, as, at certain times of the year, these vehicles were stuck on the roads and could not complete the journey to the health service. In a municipality in Matopiba, municipal ambulances remained in locations far away from the headquarters for emergency calls. In the North Minas and Semiarid regions, the car that took the team to the rural PCU could also be used for emergency transport. In the Semiarid region, another way to guarantee transport was the accreditation of private cars belonging to rural residents to transport emergency cases that could not be conveyed by the SAMU. In North Waters, there were ambulances adapted in boats – water ambulances – for crossing rivers, but they were almost always insufficient to meet the demand of the riverside population. In municipalities in the Amazon region, it was common for the health units (PCU or other health services) located in more distant and isolated areas to have transport (car or speedboat) to take users to the municipal headquarters in urgent and emergency cases.

In rare and extremely serious cases, normally in the Amazon region, air transport was used in small planes but with considerably high costs and generally hired from private companies. It was estimated that air transport had an average cost of R$15,000,00 (US$3,622) between one of the municipalities in North Waters and the location with better assistance resources.

Figure 2 summarizes the means of elective and emergency transport identified in the study by territory and the distances/time between the rural area— headquarters of the RRM—and the headquarters of the health region—the capital of the state, based on secondary data and information from managers and health professionals. It was observed that some trips in water or land vehicles exceeded 1000 km, which is more than 20 h in the North Waters and North Roads territories.

**Fig. 2:** Means of elective and emergency transport according to place of departure, distance, and estimated travel times, Remote Rural Municipalities, Brazil, 2019

## Discussion

The study results revealed that national health policies do not cover sufficient arrangements and financing to guarantee elective health transport. The policies do not cover the vast territory, the municipal asymmetries, and the numerous remote areas of the country. In the studied RRM, travel to specialized and hospital services located in other municipalities (intermunicipal flows) is frequent, but also internal travel (intramunicipal flows) so that the rural residents can access the RRM headquarters. Excessive costs and distances (which can exceed 1000 km) were found, mainly in the Amazon region. In any case, road conditions and distances are geographic and economic barriers that result in unfavorable health outcomes and inequities for residents in remote areas, findings confirmed by the primary and secondary data of this study. Thus, accessibility measurement methods and health policies that consider distance parameters combined with travel times [17] are essential in rural contexts.

Similarly, the demands for urgent and emergency transport are partially met by the SAMU important national policy [18]. Even so, there remain, in parallel, discrepancies between the federal entities in the Brazilian regions [19]. In RRM, given the diversity of territories, there is a need for availability not only of ambulances for transport (land or river), but also roads in adequate conditions of traffic, effective communication means (telephone network and internet), which implementation is dependent on intersectoral policies that integrate rural and isolated areas of Brazil.

Nevertheless, there is ample evidence suggesting that in remote settings, especially in low or middle-income countries, access to transport for health services is a resource as or more critical than the provision of health services [1, 20], implying “catastrophic expenses” [21, 22] or “financial toxicity” depending on the type of disease [5]. Expenses for travel between remote rural municipalities and the municipalities headquarters of health regions or state capitals, not provided by public resources, compromise a significant part of the families' income.

Long walks, long waiting times, or lack of public transport are factors that can turn even apparently shorter distances into barriers to the use of health services [3, 6, 8]. The unequal distribution and quality of public transport may have a more significant impact on inequalities in access to health services than spatial distribution [23]. As Porter [8] emphasizes, for low-income rural populations (off-road), whose major means of traveling is by walking, the barriers to access public health services can become insurmountable. Similarly, the elderly in rural areas, even as vehicle owners, might find it difficult to maintain and improve their quality of life when there is insufficient public transport, as the decline in car use increases with age [24]. In addition, older people are more likely to have poorer health status and limited mobility options, which can increase inequalities in access to health care and, therefore, health inequities [17].

There are multiple arrangements made by municipal managers or the users themselves to make the transport for health care possible, which are not always safe, steady, and timely. The insufficient transport for elective health service, the restriction of days, times, and routes, affects the selection of beneficiaries to socioeconomic criteria in places where vulnerability is almost always the rule. Another outcome is users not being able to attend the service, even with scheduled appointments (nonattendance) [25] and consequently causing delayed treatments and reduced time for treatment [4].

The lack of policies for the provision of transport in rural areas makes its provision dependent on insufficient municipal resources and out-of-pocket spending, which can be extremely high as show this study. If on the one hand, the municipalities provide part of the transport for health purposes, on the other hand, the municipal administration of this strategic resource without previously established criteria can favor clientelist practices. Likewise, although the resources of parliamentary amendments are relevant for the acquisition of transport in the municipalities, and indirectly represent a form of federal/state funding, it is a political resource, subject to electoral and clientelist interests, not always subject to use for local planning and reduction of inequalities in the Unified Health System [26]. To mitigate clientelist effects, one possible way is to expand the participation of organized civil society, active social movements and institutionalized social control in the formulation and implementation of programs, projects, and public policy management [27]. One of these instances is provided for in the Unified Health System legal framework, which has as one of its structuring pillars social participations through health councils and conferences (municipal, state, and national) that institutionalize the dialogue between society and the State. Paradoxically, health councils are not immune to clientelism, especially due to the asymmetry of power and knowledge among their participants and the institutional culture that can co-opt their members [28]. Another possibility to face clientelism is to give visibility, that is, to make public the problem of sanitary transport as an essential part of the care flow, which is not restricted to the provision of health services.

In addition to availability, it is not a trivial matter to consider that not everyone can drive, get a ride, or use public transport to access health services. Users with reduced mobility or with certain types of illness need adapted transport, which must be added to other alternatives such as car rental, taxis, or vouchers [4] or even reimbursement for private cars chartered by the population, as found in this study.

The result revealed high cost for health transport because of less investment in road infrastructure (unpaved roads and lack of regular public transport). The improvement of roads can optimize the distribution and transport of health supplies, a topic not addressed in this article but should also be part of the planning of the Health Care Network logistics systems [12]. The need for interconnected modes, combining different means of transport that are accessible and efficient, is even more necessary in the Amazon region, which faces the most extreme distances and costs. It is advocated that whatever the transport policy becomes, the environmental impacts should be the crucial point of any strategy, focusing on the preservation of biomes and communities, without which, there is a risk of creating or amplifying different problems [29]. In an articulated, efficient, and sustainable manner, the improvement of mobility, modes, and means increases the sense of belonging and stimulates interaction between people [8].

National policies to expand access to the internet, digital inclusion of health professionals, and rural populations is a consensual strategy for breaking physical barriers affecting access to health care [30] to connect people and territories with a positive impact on the coordination and integration of care [31]. The incorporation of telehealth, including videoconference, remote monitoring, and other modalities of remote health management, despite their disadvantages regarding doctor-patient relationships, especially among the elderly [32], are already known means for coping with geographic barriers [3]. Therefore, in a country, composed of 5,568 municipalities with continental dimensions, environmental, and socioeconomic conditions as diverse as Brazil, the low development and use of digital strategies affect the mobility of people and access to goods and services, predominantly done through water, land, and air. The disparities between municipalities due to geographic, demographic, political, technical-administrative, socioeconomic, and financial conditions show a series of problems whose confrontation extends beyond the municipal territory. In this sense, they need to be conducted and funded by the federal sphere, under strong leadership from the Ministry of Health, with a view to overcoming inequities.

It is shown that given the numerous challenges affecting transport to access health services in RRM, many of which being unresolved in the short and medium term, the real flow of users cannot be ignored. Fluvial PCU are specific modalities for PHC provision that bring assistance to riverside populations, minimizing displacements [33, 34]. The access to pharmaceutical care at home [3], mobile health units [35], eHealth interventions [36], combination and integration of telemedicine and home visits performed by health professionals [32], and continued itinerant actions, they are potentially able to provide health care closer to users and avoid displacement. Regarding access to therapeutic support, strengthening health regions so that they fulfill their role of offering, at least, specialized, and medium-complexity hospital care services, as well as the inclusion of health transport as a necessary resource for the composition of regionalized networks, which is another pending agenda in the country, would help to prevent unacceptable trips for rural populations.

Finally, given the continental dimensions of Brazil (48% of South America) and large population (6th most populous in the world), there are numerous contexts that have points in common with several Latin American countries. Many of the research findings in the Brazilian territory are like other border countries or even countries far from our borders. There are similarities between Brazil and other Latin American countries in the perspective of the low Human Development Index and vast dimensions of rural and remote territories that allow drawing analogies regarding the common challenges of access to health services and the needs of sanitary transport. In any case, any attempt to generalize and extrapolate the possible answers to the problem must always be taken in context.

### Limitations

Our findings considered the experience of health managers at various levels and PHC professionals whose perceptions and assessments were synergistic in relation to the challenges for providing elective and emergency transport in RRM, conditioned by local and regional characteristics. Experiences of other key actors, such as users, were not considered, although secondary data such as per capita income, estimated costs, and distances for the main transport modes to access health services confirm the numerous barriers faced. In any case, it is considered relevant to carry out studies at the national level that address the numerous difficulties arising from the insufficiency of public elective sanitary transport based on the experience of resident users in RRM, which is a gap between the studies developed.

## Conclusions

This study reinforces the connection between access to health transport and mitigation of the right to health care. Given the undeniable relationship between mobility and social exclusion risks due to the reduced capacity to carry out daily activities [37], it is essential to incorporate social equity criteria into the planning of transport policies. Such action also involves the availability of information on the location (latitude and longitude) of the most vulnerable families, whose mobility often occurs along unpaved side roads or paths that are not even known by public authorities and mapping platforms [11] as found in this study. It is argued that lack of policies for sufficient, continuous, and timely provision of health transport, especially for the populations that inhabit the RRM, increases the cycle of inequities and compromises the assumption of the universal right to health care.

## Data Availability

All participants provided their informed consent to participate. The data sets generated and analyzed during the current study are not publicly available due to the lack of obtained consent among the participants to share raw data. However, the data can be available upon reasonable request submitted to the corresponding author. Anonymity and confidentiality were assured according to the standard procedures, and the participants’ names and other directly identifying information were anonymized in the written text.

## Abbreviations

PCU: Primary Care Unit
RRM: Remote Rural Municipalities
PHC: Primary Health Care
IBGE: Brazilian Institute of Geography and Statistics
GDP: Gross Domestic Product
MDS: Ministry of Social Development
PBF: Bolsa Família Program
ANP: National Agency of Petroleum, Natural Gas and Biofuels
MOPS: Strategic Maps for Citizenship Policies
DER: Department of Roads and Highways
SAMU: Mobile Emergency Care Service
RM: Regional Manager
MM1: Municipal Health Secretary
MM2: PHC municipal coordinator
NUR: Nurse of the PHC team
DOC: PHC team doctor
RA: Rural area
